# Effect of geometric parameters of electrodes on skin heating for the design of non‐ablative radiofrequency device

**DOI:** 10.1111/srt.13472

**Published:** 2023-10-08

**Authors:** Yiyou Ma, Nianou Wang, Ke Li, Huan Liang, Jingfeng Bai, Xiang Ji

**Affiliations:** ^1^ School of Biomedical Engineering Shanghai Jiao Tong University Shanghai China; ^2^ Shenzhen Accompany Tech co., ltd Shenzhen China

**Keywords:** electrode design, electrothermal coupling field, non‐ablative radiofrequency skin rejuvenation, non‐ablative radiofrequency skin tightening

## Abstract

**Background:**

Non‐ablative radiofrequency (RF) has been widely used in clinical and at‐home cosmetics devices. RF electrode geometry can influence the heat distribution in the tissue. This study analyzes the influence of geometric parameters of the electrode on the heat distribution in the layered tissue.

**Materials & methods:**

The finite element simulation of the electrothermal coupling field was performed to obtain the three‐dimensional (3D) temperature distribution of the four‐layer tissue. The electrode geometric parameters including the inter‐electrode spacing (5‐12 mm), width (1‐3 mm), length (3‐10 mm), shapes (bar, dot and circle), and the coupling gel's electrical conductivity (0.2‐1.5 S/m) were simulated. The maximum temperature at 2 mm depth (*T_‐2 mm_*) and the temperature difference (*T_diff_*) between the maximum skin surface temperature and *T_‐2 mm_* were obtained to evaluate the effectiveness and safety.

**Results:**

The effect of geometric parameters on the effectiveness and safety was mixed. The maximum *T_‐2 mm_* occurred with the 5 mm inter‐electrode spacing, 3 mm width, 10 mm length, the circle‐shaped electrode, and the 1.5 S/m coupling gel's electrical conductivity. The ratio of inter‐electrode spacing to width at around four can achieve rapid temperature rise and skin surface temperature protection. The electrode shape influenced the area of temperature rise in the tissue's cross‐section. The coupling gel's electrical conductivity should be close to that of the skin to avoid energy accumulation on the skin surface.

**Conclusion:**

The electrode's geometric parameters affect the effectiveness and safety of the RF product. This study has provided the simulation procedure for the electrode design.

## 1 INTRODUCTION

In the last two decades, a great number of studies have been conducted for skin rejuvenation.^1^ Beautiful face is commonly more attractive in society, especially in the workplace.^2^ People usually pursue a good facial attractiveness to keep a positive impression. Skin rejuvenation and function repair can be achieved through several treatments. The treatments for skin rejuvenation mainly include the use of cosmetics, oral small‐molecular collagen peptides and medical cosmetology. Cosmetics protect skin from imbalances of skin function and preventing the onset of any blemishes.^3^, ^4^ However, cosmetics do not possess therapeutic properties, and they cannot fundamentally solve the problem of skin aging.^5^ The efficacy of oral administration of small‐molecule collagen peptides is unclear and few studies have demonstrated its efficacy.^6^, ^7^ Compared with these two treatments, medical cosmetology has significant advantages in its effectiveness and durability. With the enrichment and development of technology in medical cosmetology, the skin indications that can be treated are increasing.^8^ However, patients put forward more requirements for the treatments, for example, non‐invasive and painless treatment process, short recovery period after treatment, and treatment operated by the users at home.^2^ In contrast to surgery and minimally invasive treatment, physical or chemical treatments can be non‐invasive. At present, the common methods of physical and chemical therapy include laser, ultrasound, radiofrequency (RF), dermabrasion, etc.^9^ Laser is widely used in medical cosmetology including scar, facial pigmentation and facial rejuvenation.^10^, ^11^ Carbon dioxide (CO_2_) and erbium‐doped yttrium aluminum garnet (Er:YAG) lasers are the gold standards for rejuvenating photodamaged skin as non‐ablative laser systems, but their use is accompanied by a significant risk of side effects and a prolonged postoperative recovery period.^12^ Ultrasound can cause thermal damage of tissue and increase enzyme activity to repair skin function through thermal or non‐thermal mechanisms.^13^, ^14^ Dermabrasion is a form of surface remodeling and promote collagen remodeling by mechanically changing the skin at the dermal level.^15^ Dermabrasion is often accompanied by pain and its effectiveness is directly related to the manipulation of the doctor.^16^ RF therapy has few side effects and is suitable for patients with different skin types. When the high‐frequency alternating current output by the RF source flows through the skin, the particle oscillation in the tissue causes friction and generates heat due to the electrical impedance properties of skin. The thermal effect of RF leads to the contraction and deformation of collagen and induces the proliferation of new collagen, which realizes skin rejuvenation. RF has been used in medical cosmetology for more than 20 years. According to the number of electrodes or generators, RF devices are categorized into monopolar, bipolar, multipolar and multi‐source phased‐controlled.^17^, ^18^, ^19^, ^20^ Wollina performed a 20‐Caucasian‐patient open trial using the RF‐ReFacing™ device in the monopolar mode.^21^ 100% of the treated patients had an effective improvement after third treatment without adverse effects. The advantage of this type is the deep energy penetration, but it tends to accumulate the energy near the electrode on the skin surface and cause excessive temperature on the skin surface. Therefore, the skin surface should be cooled. Lee treated 26 Korean women by a bipolar RF device and obtained moderate improvements in each category of physician evaluation with limited adverse events.^22^ Palmieri ran a randomized study on 62 healthy subjects with normal‐age related‐graded skin laxity by Med‐RF^©^ device and suggested that RF significantly improves the subjective and objective judgment of patients and doctors.^23^ The electrical pathway of bipolar RF device is formed between the electrodes of different polarity and the energy penetration depth is usually half the electrode spacing.^24^, ^25^ RF energy of multipolar RF device can be split by region to avoid excessive temperature on the skin surface due to its electrode arrangement characteristics.^26^ Erkiert‐Polguj treated 30 women by multifrequency RF device (Mimari, MIP 880) and the objective evaluation in a cutometric analysis showed a statistically significant improvement between measurements taken in the pretreatment period and 3 months after the treatment.^27^ Multi‐source RF device utilizes multiple independent phased RF generators connected to an electrode array. It can generate a complex energy profile in the tissue by controlling the phase and amplitude of each generator. The repelling electrical fields result in a high temperature inside the dermal and subcutaneous layers and less heat on the epidermis.^28^, ^29^, ^30^ Tanaka evaluated the efficacy of multi‐source phase‐controlled RF.^31^ The objective assessments evaluated by a 3D color schematic representation showed improvement in skin laxity after the final treatment in all 10 patients and induced elastin appeared to be relatively thin elastic fibers without irregular elastic fibers.

Various types of RF devices have been extensively studied. However, there are few studies on the effects of electrode geometry, shape, and coupling gel on tissue energy absorption for non‐ablative RF devices. These parameters change the current density and electric field intensity in the tissue, which directly affect the RF energy absorption of the skin and then relate to the safety and efficacy of the device. Cosman and Gonzalez's clinical studies on the treatment of sacroiliac joint pain found that the lesion width could be increased to 17 and 18 mm by using a 12 and 15 mm tip spacing, respectively.^32^ Lee and Han evaluated the optimal interprobe distance for monopolar RF ablation to create large coagulation zones in the liver with the mean coagulation circularity (isometry ratio) of 0.95 ± 0.02 and 0.85 ± 0.06 at 2 and 3 cm probe spacing, respectively.^33^ Zang analyzed the effect of different electrode spacing on the electrical and thermal aspects of biological tissues during bipolar RF fat dissolution.^34^ Popa utilized a model calculation method to evaluate the energy density and electric field distribution on the models under different electric field modes of a RF applicator.^35^ The limited studies on the effect of electrode design on tissue temperature distribution resulting in the lack of theoretical guidance for the design of non‐ablative RF devices. Therefore, a simple calculation method for RF‐tissue model is needed to analyze the effects of these RF parameters on tissue temperature rise. This study provides a three‐dimensional (3D) simulation procedure of RF‐tissue electrothermal coupling model. This model can effectively calculate the spatial temperature distribution when setting different parameter values. The effects of inter‐electrode spacing, electrode width, electrode length, electrode shape, cooling/non‐cooling electrode, and coupling gel's electrical conductivity on the tissue temperature were analyzed.

## 2 METHODS

The principle of RF‐induced skin rejuvenation is an electro‐thermal coupling mechanism. When an electric current is applied to the skin, Joule heat is generated, and collagen remodeling is promoted.^36^ Electrical and thermal conduction generated by the RF electrodes on gel, skin, fat and muscle was analyzed. An electrothermal coupling model was used to obtain the RF induced 3D temperature field. The effect of RF energy on the temperature distribution was studied by varying the parameters in the simulation.

### 2.1 Electrothermal coupling model

The RF‐heating model was established based on the time domain analysis of electrothermal coupling problem.^37^ The spatial temperature distribution could be obtained by solving Pennes’ bioheat transfer equation,^38^

(1) $$\rho_{i}c_{i}\;\frac{\partial T_{i}}{\partial t}=\;\nabla \cdot \left(k_{i}\nabla T_{i}\right)+\rho_{b}c_{b}\omega_{i}\left(T_{b}-T_{i}\right)+Q_{i}+Q_{met}$$

where *ρ_i_* is the density of the tissue, *c_i_* is the specific heat of the tissue, *T_i_ ≡ T* (*x, y, z, t*) is the temperature at the position (*x, y, z*) in the Cartesian coordinate system, *t* is the time in seconds, *k_i_* is the thermal conductivity of the tissue, *ρ_b_* is the blood density, *c_b_* is the specific heat of blood, *ω_i_* is the blood perfusion rate of the tissue, *T_b_* is the blood temperature, *Q_i_* and *Q_met_* are respectively the power adsorption and metabolic heat of tissue. *Q_met_* could be ignored because of its little effect on biological heat conduction.^39^, ^40^ The sub‐index *i* represents RF gel, skin, fat or muscle, and *i =* {*g, s, f, m*}.

The rate of power adsorption per unit volume at a specific point within the tissue is proportional to the current intensity as well as the electric field intensity,

(2) $$Q_{i}=J_{i}\;\cdot \;E_{i}=\sigma_{i}\;{\left|E_{i}\right|}^{2}$$

where ***J_i_*** is the current density, *σ_i_* is the electric conductivity of the tissue, ***E_i_*** is the electrical field, which can be expressed by

(3) $$E_{i}=\;-\nabla V_{i}$$

where ***V_i_*** *≡* ***V*** (*x, y, z*) is the voltage at the position (*x, y, z*) in the Cartesian coordinate system. The quasi‐static approach is considered in the finite element model of electrothermal coupling problem since the resistive current is much lower than the displacement current. In this case, the direct current (DC) voltage applied in the model corresponds with the root mean squared (*V_rms_*) value of the RF voltage.

The heat source in this model was only produced by the RF energy, so the electric potential in the tissue was controlled by the Laplace equation given by

(4) $$\nabla \cdot \left(\sigma_{i}\nabla V_{i}\right)=\;0$$

For the part of the upper surface of RF gel without electrode coverage, natural convection with air exists according to Newton's Law of cooling as follows,

(5) $$n\cdot \;\left(k_{i}\nabla V_{i}\right)=h\left(T_{air}-T_{g}\right)$$

where ***n*** is the normal vector to the surface, *h* is the natural convection coefficient, *T_air_* is the environmental temperature, *T_g_* is the temperature at the interface between RF gel and air.

### 2.2 3D geometry of RF interaction with tissue

A 3D geometric configuration was used to simulate the RF electrodes on the skin surface with the coupling gel. The tissue was simplified to four layers including coupling gel, skin, fat and muscle. The home‐use RF device is commonly used in conjunction with the coupling gel, so the gel layer was added between the upper surface of the skin layer and RF electrodes. Both transverse and longitudinal planes of RF electrodes and the tissue layers were aligned. The details of the tissue layers and RF electrodes can be found in Figure 1. The spatial domain of this study was W×L×H, where *W* is the tissue width, *L* is the tissue length, and *H* is the depth composed of $H_{g}$, $H_{s}$, $H_{f}$ and $H_{m}$.^41^ Table 1 shows the detailed geometric parameters. The whole model was constructed using SOLIDWORKS (version 2019, Dassault Systemes Vélizy‐Villacoublay, France).

**FIGURE 1:** Configuration of tissue layers and RF electrode location with three electrode shapes. (A) Configuration of tissue layers and RF electrode, (B) bar‐shaped electrode, (C) dot‐shaped electrode, (D) circle‐shaped electrode.

**TABLE 1:** Geometric parameters of tissue layers and RF electrodes.

Parameter	Value (mm)
*W*	30
*L*	30
*H_g_*	0.5
*H_s_*	1.5
*H_f_*	3.5
*H_m_*	5
*w*	1/2/3^a^
*l_b_*	3/5/7/10^b^
*l_d_*	5
*S_b_*	5/8/10/12^c^
*S_d_*	5
*d*	2
*r_o_*	5.2
*r_i_*	4.2
*r*	2

^a^ The set of values for the electrode width.

^b^ The set of values for the electrode length.

^c^ The set of values for the inter‐electrode spacing.

### 2.3 Simulation of the tissue heated by RF energy

The simulation of RF‐induced tissue heating was performed using COMSOL Multiphysics (version 5.4, COMSOL, Burlington, MA, USA), and the resulting temperature distributions were obtained. The simulations were run on the 64‐bit server (with a dual‐processor Intel Xeon CPU E5‐2687 W v4 running at 3.00 GHz with 64 GB of RAM, Precision Tower 7910, Dell Inc.). In COMSOL Multiphysics, “LiveLink for SOLIDWORKS” function under LiveLink Interfaces sub‐node within Geometry node was used to import the 3D RF‐tissue geometry into COMSOL. Then, the corresponding material characteristics in Table 2 attached to each component were set in the material module.^42^, ^43^ Electrical properties were frequency dependent and used herein with the frequency of 1 MHz. Tissues were assumed to be isotropic materials. In the simulation, the density, heat capacity at constant pressure, thermal conductivity, electrical conductivity, permittivity and blood perfusion rate of the materials in each part of the model were constant values since variations in these parameters were not significant within the 35–45°C.^44^, ^45^, ^46^ A commercial moisturizing gel (AMIRO BEAUTY, Zongjiang Inc., Shenzhen, China) was used in the simulation and its thermal properties were measured by TEMPOS (METER Group, Inc. Pullman, WA, USA).

**TABLE 2:** Electrical and thermal parameters of different layers.

	*ε*	*σ* [S/m]	*ω* [kg/m^3^/s]	*k* [W/m/K]	*c* [J/kg/K]	*ρ* [kg/m^3^]
*Skin*	1832.8	0.22	2	0.53	3800	1200
*Fat*	27.22	0.025	0.6	0.16	2300	850
*Muscle*	1836.4	0.5	0.5	0.53	3800	1270
*Gel*	60	0.3	/	0.5	3540	1096

The electric field and thermal field were simulated using the two physical modules (“Electric Currents” and “Heat Transfer in Solids”). For bipolar RF mode (bar‐shaped electrode and circle‐shaped electrode), one of the RF electrodes were modeled as a constant‐voltage source and the other one was set as “Ground” condition. For the dot‐shaped electrodes, the three left electrodes were modeled as the same voltage source while the three right ones were set as “Ground” condition. Zero electric flux condition was considered at the residual coupling gel surface, the bottom area of the muscle layer and the axial boundaries.^47^ “Terminal” boundary module was used in the “Current” module to set the constant voltage on each electrode part.

In the Heat Transfer in Solids module, the initial temperature of the electrodes and the tissue was set in the “Initial Values” boundary condition. The natural convection of the coupling gel was simulated by the “Heat Flux” boundary condition. The heat loss by blood perfusion of the skin, fat, and muscle were set in “Biological Tissue” boundary condition. Zero heat flux condition was considered at the bottom area of the muscle layer and the axial boundaries. The initial temperature boundary conditions are shown in Table 3.

**TABLE 3:** Initial temperature boundary conditions.

Parameter	Value (units)
*T_air_*	293.15 (K)
*T_b_*	310.15 (K)
*T_c_*	293.15 (K)
*h*	10 (W/m^2^/K)

Normal size of physics‐controlled mesh in the sequence type was chosen with the consideration of computation time, and the higher mesh density showed in the RF electrodes and coupling gel. The time step was 1 s, and the 3D temperature field was simulated with 20 s of RF heating under different setting parameters.

### 2.4 Efficacy and safety evaluation

The home‐use RF device can be used to elevate the subcutaneous tissue temperature to the setting temperature in a short period (i.e., 42°C in 20 s), and the collagen can be improved after maintaining this temperature for a period of time.^41^, ^48^ Therefore, the maximum temperature of the subcutaneous tissue at 2 mm depth (*T_‐2 mm_*) after 20 s operation time of the RF device was selected in this study, while the effective temperature was selected as 42°C.^49^ Besides, the skin safety is also another consideration for the device because of its special home‐use scenario. To avoid skin burning, the skin surface temperature should be kept at no more than 45°Cduring the operation period.^50^ In this study, the temperature difference (*T_diff_*) between the maximum skin surface temperature (*T_s_*) and *T_‐2 mm_* was selected for safety evaluation. Within the safe temperature threshold, a smaller *T_diff_* indicates better safety and effectiveness because *T_‐2 mm_* is higher. The temperature results (*T_s_, T_‐2 mm_*, *T_diff_*) of different RF electrode shapes and the 2D temperature distribution at 2 mm under the skin were obtained. In this study, the heat at different tissue depths were observed from temperature distribution in longitudinal section.

Power density was used to quantify the RF energy absorbed by tissues.^17^, ^24^ High power density gives rise to the high heat absorption.^34^, ^47^ Power density is determined by both current density and electric field intensity (Equation 2). Therefore, current density and electric field intensity were used to analyze the temperature difference.

### 2.5 Design factors of the home‐use RF device

The electrode structure and power setting are important for the design of the home‐use RF device because they can greatly affect the product performance. In addition, the electrical conductivity of the RF coupling gel can change the heat distribution of the tissue by influencing the electric field. Therefore, the design factors in this study included the electrode geometric parameters, electrode shape, the electrode with or without cooling and electric conductivity of the coupling gel. In the electrode geometric parameters, electrode width, inter‐electrode spacing and electrode length were analyzed in detail. In the analysis of the influence of electrode geometric parameters on the tissue temperature, the electrode widths were 1 mm, 2 mm, and 3 mm. The inter‐electrode spacing were 5 mm, 8 mm, 10 and 12 mm. The electrode lengths were 3 mm, 5 mm, 7 and 10 mm, respectively. The bar‐shaped, dot‐shaped and circle‐shaped electrodes were used since the aforementioned three shapes of electrodes cover most of the electrode shapes of the current RF devices.^51^ The maximum contour area of each electrode combination was designed to be the same to ensure the comparability of results of electrodes with different shapes (*S_d_* = 5 mm, *w* = 2 mm, *r_o_* = 5.2 mm). Meanwhile, the area ratio of a positive electrode and negative electrode was 1 to avoid the area effect of electrodes with different polarity. The electrode temperature was set to 20°C during the whole operation period as the cooling mode to analyze its effect on the temperature distribution while the electrode temperature without limitation was considered as non‐cooling mode. In the analysis of the gel conductivity, the values were set at 0.2, 0.6, 1.0, and 1.5 S/m. It was assumed to be an isotropic material in the simulation, and the density, heat capacity at constant pressure, thermal conductivity, electrical conductivity, permittivity and blood perfusion rate of the materials in each part of the model did not change with the possible temperature elevation.

## 3 RESULT

### 3.1 Geometric parameters of RF electrodes

#### 3.1.1 Inter‐electrode spacing

Table 4 shows the temperatures of *T_s_, T_‐2 mm_*, *T_diff_* at different voltages (20 V, 30 V, 40 V) with the inter‐electrode spacing of 5 mm, 8 mm, 10 and 12 mm. As the spacing was changed from 5 to 12 mm, the *T_s_* was decreased from 39.8°C to 35.2°C (20 V), 48.0°C to 37.6°C (30 V), 59.4°C to 41.1°C (40 V), respectively. *T_‐2 mm_* was decreased from 38.1°C to 35.6°C (20 V), 42.4°C to 36.7°C (30 V), 48.5°C to 38.3°C (40 V). *T_diff_* decreased from 1.7°C to −0.4°C (20 V), 5.5°C to 0.9°C (30 V), and 10.9°C to 2.8°C (40 V). For the different inter‐electrode spacings at the same voltage, *T_‐2 mm_* and *T_diff_* were the highest with the inter‐electrode spacing of 5 mm. In addition, Figure 2 demonstrates that the deepest depth and the largest area of temperature elevation were achieved for the 5 mm inter‐electrode spacing, whereas *T_‐2 mm_* and *T_diff_* were the lowest for the inter‐electrode spacing of 12 mm, and the depth with the effective temperature elevation was least and the area was smallest.

**TABLE 4:** Simulation results of different inter‐electrode spacings.

Voltage [V]	*W* [mm]	*S_b_* [mm]	*T_s_* [°C]	*T_‐2 mm_* [°C]	*T_diff_* [°C]
20	2	5	39.8	38.1	1.7
	2	8	36.2	36.2	−0.1
	2	10	35.6	35.8	−0.2
	2	12	35.2	35.6	−0.4
30	2	5	48.0	42.4	5.5
	2	8	38.9	38.2	0.7
	2	10	38.5	37.2	1.3
	2	12	37.6	36.7	0.9
40	2	5	59.4	48.5	10.9
	2	8	45.1	41.0	4.1
	2	10	42.6	39.2	3.4
	2	12	41.1	38.3	2.8

**FIGURE 2:** Temperature distribution of different inter‐electrode spacings with the same electrode width at different voltages for 20 s (In each row, the voltage value corresponding to the results from left to right is 20 V, 30 V and 40 V, respectively. The inter‐electrode spacing from top to bottom in each row is 5 mm, 8 mm, 10 and 12 mm, respectively). (A) Temperature distribution in longitudinal section, (B) Temperature distribution of 2 mm cross‐section under the skin surface.

**FIGURE 3:** *T_‐2 mm_* and *T_diff_* of different inter‐electrode spacings with the same electrode width.

#### 3.1.2 Electrode width

Table 5 shows the *T_s_, T_‐2 mm_*, *T_diff_* of the electrode widths (1 mm, 2 and 3 mm) at different voltages. As the width was changed from 1 to 3 mm, the *T_s_* was increased from 38.4°C to 42.4°C (20 V), 44.9°C to 53.9°C (30 V), 53.8°C to 70.2°C (40 V), respectively. The *T_‐2 mm_* was increased from 37.1°C to 39.1°C (20 V), 40.2°C to 44.7°C (30 V), 44.5°C to 52.5°C (40 V). The *T_diff_* was increased from 1.3°C to 3.3°C (20 V), 4.7°C to 9.3°C (30 V), 9.4°C to 17.6°C (40 V). For the different electrode widths at the same voltage, the *T_‐2 mm_* and *T_diff_* were the highest with the electrode width of 3 mm. Figure 4 demonstrates that the deepest depth and the largest area shown of the temperature elevation were achieved for the 3 mm electrode width, whereas the electrode width was 1 mm, the *T_‐2 mm_* and *T_diff_* were lowest along with the lowest depth and the smallest area of the temperature elevation.

**TABLE 5:** Simulation results of different electrode widths.

Voltage [V]	*W* [mm]	*S_b_* [mm]	*T_s_* [°C]	*T_‐2 mm_* [°C]	*T_diff_* [°C]
20	1	5	38.4	37.1	1.3
	2	5	39.8	38.1	1.7
	3	5	42.4	39.1	3.3
30	1	5	44.9	40.2	4.7
	2	5	48.0	42.4	5.5
	3	5	53.9	44.7	9.3
40	1	5	53.8	44.5	9.4
	2	5	59.4	48.5	10.9
	3	5	70.2	52.5	17.6

**FIGURE 4:** Temperature distribution of the same inter‐electrode spacing, different electrode width and different voltage values at 20 s (In each row, the voltage value corresponding to the results from left to right is 20 V, 30 V and 40 V, respectively. The electrode width from top to bottom in each row is 1 mm, 2 and 3 mm, respectively). (A) Temperature distribution in longitudinal section. (B) Temperature distribution of 2 mm cross‐section under the skin surface.

**FIGURE 5:** The *T_‐2 mm_* and *T_diff_* of different electrode widths with the same inter‐electrode spacing.

#### 3.1.3 Electrode length

Table 6 shows the *T_s_, T_‐2 mm_*, *T_diff_* of the four electrode lengths (3 mm, 5 mm, 7 and 10 mm) at different voltages. As the length was changed from 3 to 10 mm, the *T_s_* was increased from 39.6°C to 39.8°C (20 V), from 47.4°C to 48.0°C (30 V), from 58.4°C to 59.4°C (40 V), respectively. The *T_‐2 mm_* was increased from 37.4°C to 38.1°C (20 V), from 40.9°C to 42.4°C (30 V), and from 45.7°C to 48.5°C (40 V). The *T_diff_* was decreased from 2.1°C to 1.7°C (20 V), 6.6°C to 5.5°C (30 V) and 12.7°C to 10.9°C (40 V). For the different electrode lengths at the same voltage, the *T_‐2 mm_* was highest while the *T_diff_* was the lowest with the electrode length of 10 mm. In addition, Figure 6 also demonstrates that the largest area of the temperature elevation was achieved for the 10 mm electrode length, but no significant difference of the depth with the temperature elevation was observed at 40 V. Whereas the *T_‐2 mm_* was lowest and the *T_diff_* was highest for the 3 mm electrode length, and the area of the temperature elevation was also smallest.

**TABLE 6:** Simulation results of different electrode lengths.

Voltage [V]	*W* [mm]	*S_b_* [mm]	*l_b_* [mm]	*T_s_* [°C]	*T_‐2 mm_* [°C]	*T_diff_* [°C]
20	2	5	3	39.6	37.4	2.1
	2	5	5	39.6	37.6	2.0
	2	5	7	39.7	38.0	1.7
	2	5	10	39.8	38.1	1.7
30	2	5	3	47.4	40.9	6.6
	2	5	5	47.6	41.2	6.4
	2	5	7	47.8	42.3	5.5
	2	5	10	48.0	42.4	5.5
40	2	5	3	58.4	45.7	12.7
	2	5	5	58.8	46.2	12.6
	2	5	7	59.2	48.4	10.8
	2	5	10	59.4	48.5	10.9

**FIGURE 6:** Temperature distribution of different electrode lengths (area) and different voltage values at 20 s (In each row, the voltage value corresponding to the results from left to right is 20 V, 30 V and 40 V, respectively. The electrode length from top to bottom in each row is 3 mm, 5 mm, 7 and 10 mm, respectively). (A) Temperature distribution in longitudinal section. (B) Temperature distribution of 2 mm cross‐section under the skin surface.

**FIGURE 7:** The *T_‐2 mm_* and *T_diff_* of different electrode lengths.

#### 3.1.4 Electrode shape

Table 7 shows the *T_s_, T_‐2 mm_*, *T_diff_* of the bar‐shaped, dot‐shaped and circle‐shaped electrodes at different voltages. With the voltage set at 20 V, the *T_s_* were 39.8°C, 40.4°C and 52.4°C, respectively for the bar‐shaped, dot‐shaped and circle‐shaped electrodes; the *T_‐2 mm_* was 38.1°C, 37.9°C and 41.2°C, and the *T_diff_* was 1.7°C, 2.5°C and 11.2°C. More detailed results can be found in Table 7. At the same voltage, both the deepest depth and the largest area of the temperature elevation were achieved for the circle‐shaped electrode (see Figure 8). The similar depths of the temperature elevation were achieved in the dot‐shaped electrode and bar‐shaped electrode, but the area of the temperature elevation was smallest for the dot‐shaped electrode.

**TABLE 7:** Simulation results of different electrode shapes.

Voltage [V]	Electrode shape	*T_s_* [°C]	*T_‐2 mm_* [°C]	*T_diff_* [°C]
20	Bar	39.8	38.1	1.7
	Dot	40.4	37.9	2.5
	Circle	52.4	41.2	11.2
30	Bar	48.0	42.4	5.5
	Dot	49.3	42.0	7.3
	Circle	76.2	49.2	27.0
40	Bar	59.4	48.5	10.9
	Dot	61.8	47.7	14.1
	Circle	109.6	60.5	49.1

**FIGURE 8:** Temperature distribution of the same ratio of the maximum contour area of the electrode and cross‐section area of tissue at 20 s (In each row, the voltage value corresponding to the results from left to right is 20 V, 30 V and 40 V, respectively. The electrode shape from top to bottom in each row is bar‐shaped, dot‐shaped and circle‐shaped, respectively). (A) Temperature distribution in longitudinal section. (B) Temperature distribution of 2 mm cross‐section under the skin surface.

### 3.2 Electrical conductivity of coupling gel

Table 8 shows the *T_s_, T_‐2 mm_* and *T_diff_* with four electrical conductivities of the RF coupling gel (0.2 S/m, 0.6 S/m, 1.0 S/m and 1.5 S/m) at different voltages. As the electrical conductivity was changed from 0.2 S/m to 1.5 S/m, the *T_s_* was increased from 39.8°C to 62.4°C (20 V), 48.0°C to 98.8°C (30 V), 59.4°C to 149.9°C (40 V), respectively. The *T_‐2 mm_* was increased from 38.1°C to 45.3°C (20 V), 42.4°C to 58.6°C (30 V), 48.5°C to 77.3°C (40 V). The *T_diff_* was decreased from 1.7°C to 17.1°C (20 V), 5.5°C to 40.2°C (30 V), 10.9°C to 72.7°C (40 V). For the different electrical conductivities at the same voltage, the *T_‐2 mm_* and *T_diff_* were highest with the electrical conductivity of 1.5 S/m. And the deepest depth and the largest area of the temperature elevation were also achieved for the 1.5 S/m electrical conductivity (see Figure 9). When the electrode spacing is 0.2 S/m, both the *T_‐2 mm_* and *T_diff_* were lowest for the 0.2 S/m electrical conductivity, and the lowest depth and the smallest area were achieved.

**TABLE 8:** Simulation results with different electrical conductivities of the gel.

Voltage [V]	*W* [mm]	*S_b_* [mm]	Electrical conductivity (S/m)	*T_s_* [°C]	*T_‐2 mm_* [°C]	*T_diff_* [°C]
20	2	5	0.2	39.8	38.1	1.7
	2	5	0.6	47.1	40.7	6.4
	2	5	1.0	53.9	42.8	11.1
	2	5	1.5	62.4	45.3	17.1
30	2	5	0.2	48.0	42.4	5.5
	2	5	0.6	64.4	48.2	16.2
	2	5	1.0	79.8	53.0	26.9
	2	5	1.5	98.8	58.6	40.2
40	2	5	0.2	59.4	48.5	10.9
	2	5	0.6	88.7	58.8	29.8
	2	5	1.0	116.1	67.2	48.8
	2	5	1.5	149.9	77.3	72.7

**FIGURE 9:** Temperature distribution of different electrical conductivities of RF gel at 20 s (In each row, the voltage value corresponding to the results from left to right is 20 V, 30 V and 40 V, respectively. The electrical conductivity from top to bottom in each row is 0.2 S/m, 0.6 S/m, 1.0 S/m and 1.5 S/m, respectively). (A) Temperature distribution in longitudinal section. (B) Temperature distribution of 2 mm cross‐section under the skin surface.

**FIGURE 10:** The *T_‐2 mm_* and *T_diff_* of different electrical conductivities.

## 4 DISCUSSION

The electric field intensity and current density influence the energy absorption into the tissue.^34^ While they are determined by the electrode geometry, shape and electrical conductivity of RF coupling gel, which are of great importance to the temperature distribution in the tissue. The gradient of the temperature change curve in the figure results (Figures 3, 5, 7, 10) is represented as the temperature change rate.

### 4.1 Effect of electrode geometric parameters on temperature distribution

The simulation temperature results of the electrode geometric parameters have illustrated that the inter‐electrode spacing and electrode width would greatly influence the temperature distribution of the skin. As the inter‐electrode spacing was increased or the electrode width was decreased, both *T_‐2 mm_* and *T_diff_* were decreased. The temperature change rate slowed down with the increase of electrode spacing (see Figure 3), but accelerated with the increase of electrode width (see Figure 5). Figures 2 and 4 have demonstrated that the 5 mm electrode spacing and the 3 mm electrode width have the deepest effective temperature depth and the largest coverage volume, respectively. Thus, smaller inter‐electrode spacing or larger electrode width could achieve the faster temperature rise. In addition, the temperature elevation in 20 s was not obvious with the more than 10 mm inter‐electrode spacing (see Figure 3). It's because the energy absorbed by the tissue was offset by the heat dissipation of the RF gel.

The electrode width could change the spacing between the inter‐electrode edges. As the electrode width was increased, the edge spacing between the two electrodes was decreased and it could cause the increase of the electric field intensity on the gel surface. The increase in electric field intensity led to energy aggregation which increased *T_diff_*. There was a significant correlation between the inter‐electrode spacing and electrode width so these two parameters jointly affected the temperature distribution. Therefore, in order to explore the joint effect of both inter‐electrode spacing and electrode width on the temperature distribution, the ratio of the electrode spacing to the electrode width was considered as the new design parameter of electrodes. *T_s_, T_‐2 mm_* and *T_diff_* were decreased when the ratio was increased from 1.67 to 6. Figure 11 has demonstrated that the temperature was stable when the ratio value was higher than 4, and the details results can be found in Table 9.

**FIGURE 11:** *T_‐2 mm_* and *T_diff_* versus the ratio of inter‐electrode spacing to the electrode width.

**TABLE 9:** Temperatures with different values of the ratio of the inter‐electrode spacing to the electrode width.

Voltage [V]	*W* [mm]	*S_b_* [mm]	Ratio	*T_s_* [°C]	*T_‐2 mm_* [°C]	*T_diff_* [°C]
20	3	5	1.67	42.4	39.1	3.3
	2	5	2.5	39.8	38.1	1.7
	2	8	4	36.2	36.2	−0.1
	2	10	5	35.6	35.8	−0.2
	2	12	6	35.2	35.6	−0.4
30	3	5	1.67	53.9	44.7	9.3
	2	5	2.5	48.0	42.4	5.5
	2	8	4	38.9	38.2	0.7
	2	10	5	38.5	37.2	1.3
	2	12	6	37.6	36.7	0.9
40	3	5	1.67	70.2	52.5	17.6
	2	5	2.5	59.4	48.5	10.9
	2	8	4	45.1	41.0	4.1
	2	10	5	42.6	39.2	3.4
	2	12	6	41.1	38.3	2.8

Longer electrode length can greatly enlarge the area of the skin covered by the electrodes, but has little effect on the effective depth of the temperature elevation. Figure 7 has demonstrated that the increase in the electrode length resulted in the little increase in *T_‐2 mm_* and little decrease in *T_diff_*. The change in the electrode length did not change the electrode width and inter‐electrode spacing, so the electric field intensity and current density were barely affected. Although the varied electrode length altered the energy distribution area, there was no significant change in *T_‐2 mm_* (see Table 6).

In the three types of electrode shapes, *T_‐2 mm_* and *T_diff_* of the circle‐shaped electrode were the highest. Besides, Figure 8 shows that the circle‐shaped electrode also had the deepest penetration depth of effective temperature and fastest temperature rise rate (see in Table 7). The heat penetration depth of the dot‐shaped electrode was comparable to that of the bar‐shaped electrode, but the heat generated by dot‐shaped electrodes covered the smaller area. The bar‐shaped electrode would be safer for the skin because the smallest temperature difference between the skin surface and −2 mm deep skin was achieved. Different electrode shapes had direct influence on the temperature distribution and penetration depth, which might be the different energy coverage area and distribution of the tissue caused by the variational intensities of electric field in the skin.

The effect of the electrode area on the skin temperature depends on the geometric parameters of electrodes. The increase in the width or length of the electrodes can enlarge the electrode area, but the two geometric parameters of electrodes have the different effects on the skin temperature rise. For the different shapes of electrodes with the same inter‐electrode spacing and width (diameter for dot‐shaped electrodes), the bar‐shaped electrode had a larger electrode area than that of dot‐shaped electrodes. The *T_‐2 mm_* of the bar‐shaped electrode was higher than that of the dot‐shaped electrode, while the *T_diff_* of the former was lower than that of the latter. The current density around the dot‐shaped electrode was larger at the same voltage because of its relatively small electrode area. The high current density would produce more energy absorption in the gel or the skin around the electrode and it would result in the larger temperature difference. Therefore, for the same inter‐electrode spacing and electrode width, the increase in the electrode area can avoid excessive current density and reduce the temperature difference.

The coupling gel is used to couple the electrode and the skin and its electrical conductivity could directly reflect in the energy absorption of skin. When the coupling gel's electrical conductivity was increased, both *T_s_* and *T_‐2 mm_* were significantly increased. The *T_diff_* was also increased with the increase of coupling gel's electrical conductivity, and the linear positive correlation was observed between the *T_diff_* and electrical conductivity. It was found that *T_diff_* increased faster than the *T_‐2 mm_* (see Figure 10) because the current density of the gel layer and the skin surface is higher. The coupling gel with the high electrical conductivity may not be selected due to the safety concern caused by the fast temperature rise on the skin surface. Therefore, the electrical conductivity of coupling gel should be considered in the design of the electrodes’ geometric parameters for safety.

### 4.2 Effect of cooling/non‐cooling electrode on temperature distribution

For all combinations with the same settings except cooling or non‐cooling electrodes, the results of electrical conductivity with 0.2 S/m and the electrode voltage with 40 V are shown below. For the electrodes in the cooling mode, *T_s_*, *T_‐2 mm_* and *T_diff_* were decreased significantly. However, Table 10 demonstrates that *T_s_* was still higher than *T_‐2 mm_*. Figures 12, 13, 14 show that the area and depth of effective temperature elevation were greatly decreased for the cooling electrodes. Besides, in the cooling mode, the *T_diff_* could be also reduced to improve safety. The main limitation of the cooling electrode is that the cooling effect would reduce the heat absorbed by the skin so that the skin temperature rise rate and heating area are decreased.

**TABLE 10:** Results of cooling/non‐cooling electrodes with DC = 40 V.

	*W* [mm]	*S_b_* [mm]	*S_b_* [mm]	*T_electrode_* [°C]	*T_s_* [°C]	*T_‐2 mm_* [°C]	*T_diff_* [°C]
Spacing	2	5	10	/	59.4	48.5	10.9
	2	5	10	20	49.4	44.2	5.2
	2	8	10	/	45.1	41.0	4.1
	2	8	10	20	41.5	39.8	1.7
	2	10	10	/	42.6	39.2	3.4
	2	10	10	20	38.7	38.1	0.6
Width	1	5	10	/	53.8	44.5	9.4
	1	5	10	20	44.7	41.5	3.2
	3	5	10	/	70.2	52.5	17.6
	3	5	10	20	53.8	46.3	7.5
Length	2	5	3	/	58.4	45.7	12.7
	2	5	3	20	46.6	41.5	5.1
	2	5	5	/	58.8	46.2	12.6
	2	5	5	20	48.1	42.5	5.7
	2	5	7	/	59.2	48.4	10.8
	2	5	7	20	48.9	43.5	5.4

**FIGURE 12:** Temperature distribution of cooling/non‐cooling electrodes with two inter‐electrode spacings (5 and 8 mm) and different voltages for the 20 s operating period. (A) Temperature distribution in longitudinal section. (B) Temperature distribution of 2 mm cross‐section under the skin surface (* represents cooling electrodes).

**FIGURE 13:** Temperature distribution of cooling/non‐cooling electrodes with two electrode widths (1 mm an 3 mm) and different voltages for the 20 s operation period. (A) Temperature distribution in longitudinal section. (B) Temperature distribution of 2 mm cross‐section under the skin surface (* represents cooling electrodes).

**FIGURE 14:** Temperature distribution of cooling/non‐cooling electrodes with two electrode lengths (3 and 7 mm) and different voltages for the 20 s operation period. (A) Temperature distribution in longitudinal section. (B) Temperature distribution of 2 mm cross‐section under the skin surface (* represents cooling electrodes).

### 4.3 Design case

This study has provided the parameter analysis of the electrode geometry and the selection of the coupling gel for the design of the home‐use RF device. Based on the simulated result of geometric parameters, a new design using the bar‐shaped RF electrode was given below. According to the Figure 11, the ratio of the inter‐electrode spacing to the electrode width was set at 4 for the safety and temperature elevation in the 2 mm depth. Optionally, the electrode width was 1 mm and the inter‐electrode spacing was 4 mm. Six electrodes were arranged with alternated positive and negative electrodes (see Figure 15). The electrode length can be increased in an adjustable range and was set to 20 mm in this design. The coupling gel's electrical conductivity could be slightly less than that of the skin, and the value was set as 0.2 S/m. The cooling mode of the electrode was selected to protect the skin surface. In this design, the increase in the electrode number can expand the area of the skin surface covered by the electrodes and the area of the temperature rise on the skin surface under the electrode was significantly enlarged (see Figure 16). With the voltage of 40 V, the maximum *T_‐2 mm_* reached 42.5°C and the maximum *T_diff_* was 5.2°C, which was also in the safe profile. The above procedure can be used for the electrode design and the iteration of the existing electrodes. In addition, different shapes of electrodes can be also combined to achieve the specific design purpose.

**FIGURE 15:** Electrode polarity setting.

**FIGURE 16:** Temperature distribution of the design case. The upper row is the temperature profiles on the 2 mm deep under the skin surface and the bottom row is the temperature profiles in longitudinal section.

In the electrode design of the home‐use RF device, operation safety and efficacy should be considered, and the aesthetics is also of great importance for the marketing demand. This study has provided the simulated results of the temperature distribution from different design parameters of electrode geometry, and the associated parameter analysis of the effects of the geometric parameters and gel's electrical conductivity on the temperature distribution could be helpful for the concept design.

The electrodes of the home‐use RF devices are generally bipolar or multipolar electrodes. The direction of the generated electric field is not perpendicular to the skin, which makes the epidermis and dermis absorb more energy so that the temperature of the skin surface rise faster than that of the subcutaneous fat. The cooling protection of the skin surface is used to avoid the skin burns during the treatment process as well as reduce the pain.^52^ In the clinical application, local anesthesia and epidermis pre‐cooling are usually used to relieve pain and reduce the temperature of the epidermis, respectively.^53^ In the ThermaCool (Thermage Inc., Hayward, CA, USA), a concurrent spray of cryogen spares are applied on the back of the electrode to protect the epidermis.^54^ But this cooling technology is not suitable for the home use due to the limited space and cost. The coupling gel owns good thermal conductivity and heat dissipation characteristics, and it also has the good performance both in current conduction and skin surface heat dissipation. The simulated results shown in Figure 16 and Table 11 have demonstrated that the temperature on the skin surface were still higher than that in the subcutaneous fat with coupling gel. The temperature difference can be reduced by appropriately increasing the thickness of the coupling gel. Alvaro also mentioned a temperature‐controlling multipolar handpiece which could be applied to a sequence of electrical modulation to avoid tissue overheating.^55^ The skin surface cooling is a key point to improve the safety and efficacy of home‐use RF devices. Therefore, the small cooling module and electrical modulation will be integrated into the home‐use RF device in future.

**TABLE 11:** Simulated results of the design case.

Voltage (V)	*T_s_* [°C]	*T_‐2 mm_* [°C]	*T_diff_* [°C]
20	33.5	35.3	−1.8
30	39.4	38.1	1.3
40	47.7	42.5	5.2

## 5 CONCLUSION

The simulation of the electrothermal coupling field between RF and four‐layer tissue has been performed to obtain the 3D temperature distribution of the tissue. The simulated results have demonstrated that the geometric parameters of the electrode (inter‐electrode spacing, width, length, shape) and the coupling gel's electrical conductivity have significant effects on the temperature distribution of the tissue. With the ratio of inter‐electrode spacing to width set at about 4, the rapid tissue temperature rise and skin surface protection can be achieved. Electrode length could not significantly change the *T_diff_*. And the selection of an optimal electrode shape can effectively enlarge the area of temperature rise in the cross section of the covering tissue. The electrical conductivity of the selected coupling gel should be close to that of the skin to avoid the massive energy flowing through the coupling gel to the skin surface. The cooling electrode can effectively reduce the *T_diff_*. In the design of the RF device, the appropriate geometric parameters of the electrodes play an important role in the effectiveness and safety of the product, and this study has provided the simulation procedure for the electrode design.

## CONFLICT OF INTEREST STATEMENT

The authors declare no conflicts of interest.

## Data Availability

The data that support the findings of this study are available from the corresponding author upon reasonable request.
